RETRACTED

# Ultrasound versus temporal artery biopsy in patients with Giant cell arteritis: a prospective cohort study

**DOI:** 10.1186/s12880-019-0344-2

**Published:** 2019-06-06

**Authors:** Quan Zou, Sumei Ma, Xinghu Zhou

**Affiliations:** 1 Department of Ultrasound, the first hospital of Lanzhou University, Lanzhou, 730000 China; 2 Department of Cardiology, the first hospital of Lanzhou University, Lanzhou, 730000 China

**Keywords:** Giant cell arteritis, Magnetic resonance imaging, Overdiagnosis, Overtreatment, Temporal artery biopsy, Ultrasound

## Abstract

**Background:**

Diagnosis of giant cell arteritis by temporal artery biopsy is time-consuming and visual loss lies in the first week after its diagnosis. The purpose of the study was to test the hypothesis that ultrasound can reduce the risk of overdiagnosis and overtreatment in giant cell arteritis.

**Methods:**

Data regarding physical/ clinical features examinations, temporal artery biopsy examinations, ultrasound findings, and magnetic resonance imaging examinations of 980 suspected patients for giant cell arteritis were included in the study. Decision curve analysis was applied to get a beneficial score for selected diagnostic modalities. Cost analysis was performed for each patient.

**Results:**

Fewer numbers of false positive giant cell arteritis results were reported under physical/ clinical features examinations following ultrasound detection than physical/clinical features examinations following temporal artery biopsy examinations (45 vs. 127, *p* < 0.0001). The working area that detects giant cell arteritis at least one time for physical/ clinical features examinations following ultrasound detection and physical/ clinical features examinations following temporal artery biopsy examinations were 0–91% and 0–86%. No significant difference for true negative results between magnetic resonance imaging and physical and clinical features examinations following ultrasound detection (*p* = 0.007). Physical and clinical features examinations following ultrasound detection were less expensive method than physical/ clinical features examinations following temporal artery biopsy examinations (14,023 ± 982 ¥/patient vs. 18,551 ± 1231 ¥/patient, *p* < 0.0001) and MRI.

**Conclusion:**

Physical and clinical features examinations following ultrasound are recommended for diagnosis of patients with suspected giant cell arteritis.

## Background

Giant cell arteritis or temporal arteritis is vasculitis and has been found in more than 50 years age people [1] leads to aortitis, stroke, blindness [2], or myocardial infarction [3]. Very large populations with giant cell arteritis are found in China [4]. Glucocorticoid treatment after rapid diagnosis is generally recommended in giant cell arteritis [5]. The diagnosis of giant cell arteritis is not straightforward but it is made on temporal artery biopsy and the decision is supported by presenting symptoms [6] but its sensitivity is varied from 39 to 91%, because of drug intake e.g. glucocorticoid took by patients have effect on the results of temporal artery biopsy means, has large numbers of false negatives results can be found [1], which lead to use of a high dose of glucocorticoid as precaution. Moreover, diagnosis by temporal artery biopsy is time-consuming [7] and visual loss lies in the first week after its diagnosis [8]. In short, temporal artery biopsy is considered as ‘gold standard’ for giant cell arteritis [9] but there are poor associations between the results of temporal artery biopsy and giant cell arteritis especially multi-vessels giant cell arteritis [10]. Besides, temporal artery biopsy, ultrasound [11] and magnetic resonance imaging (MRI) [12] are non-invasive techniques used for diagnosis of giant cell arteritis but MRI has issues of availability and cost [1]. Additionally, no ionizing radiation involved in ultrasound [13]. Ultrasound has high specificity (100%) but very low (43%) sensitivity was reported for the diagnosis of giant cell arteritis [14]. Moreover, glucocorticoid treatment can be started before a formal diagnosis, which leads to weight gain, hypertension, cataract, osteoporosis, and thin skin [1]. Overall, giant cell arteritis has problems of overdiagnosis and overtreatment.

RETRACTED

The primary aim of the study was to compare sensitivity, specificity, and cost of ultrasound with temporal artery biopsy considering MRI as a reference standard in patients with suspected giant cell arteritis. The secondary endpoint of the study was to test the hypothesis that ultrasound can reduce the risk of overdiagnosis and overtreatment in giant cell arteritis.

## Methods

### Reagents

Formalin, glycerin, hematoxylin, and eosin were purchased from Mark Specialist Pvt. Ltd., Berlin, Germany. Gadolinium (Omniscan) was purchased from GE Healthcare, Salt Lake City, Utah, USA.

### Inclusion criteria

Patients with recent visual impairment, C-reactive protein level less than 5 mg/dL, jaw or tongue claudication, shoulder girdles (pain and stiffness in the shoulder), pain in the hip (pelvic girdles), abnormal liver functions, or temporal artery tenderness referred by rheumatologists, ophthalmologist, and neurologists (all have minimum 3-years’ experience) to the hospital were included in the study cohort.

### Exclusion criteria

Patients with known giant cell arteritis were excluded from the study. Patients who had to receive glucocorticoid treatment (any glucocorticoid treatment less than 6-months prior to study) for the other reason(s) were excluded from enrollment.

RETRACTED

### Physical and clinical features examinations

The evidence of thickening, tenderness, and pulsation of both axillary arteries, scalp, and tongue necrosis were physically examined by neuro physicians (minimum 3-years’ experience, blinded regarding clinical examinations, temporal artery biopsy examinations, ultrasound examinations, and MRI examinations) of the institute. The evidence of posterior or anterior ischemic optic neuropathy, afferent pupillary defect, III/IV/V nerve palsy or bruits on either side were examined by ophthalmologists (minimum 3-years’ experience, blinded regarding clinical examinations, temporal artery biopsy examinations, ultrasound examinations, and MRI examinations) of the institute. The evidence of stroke and aneurysm were examined by a physician (minimum 3-years’ experience, blinded regarding clinical examinations, temporal artery biopsy examinations, ultrasound examinations, and MRI examinations) of the institutes. The sample of blood was collected from each patient and send to a laboratory for examinations of erythrocyte sedimentation rate (ESR), C-reactive protein level, plasma viscosity, blood cell counts, and hemoglobin. All pathological examinations had been made by pathologists (minimum 3-years’ experience, blinded regarding physical features, temporal artery biopsy examinations, ultrasound examinations, and MRI examinations) of the institute [1]. If age at least 50 years, temporal artery abnormalities, elevated ESR (≥ 50 mm/h), the new type of localized head pain, and claudication of jaw or tongue was reported in the patient then it was considered as giant cell arteritis [5].

### Temporal artery biopsy examinations

The one-centimeter temporal artery was collected from patients by surgical procedure and send to the laboratory of the institute. The sample was fixed in formalin, embedded in a paraffin block, and slides were stained with hematoxylin and eosin. The prepared slides were observed under a light microscope (Olympus, Beijing, China) in 100 magnifications (Fig. 1) [11]. Histopathological examinations had performed by pathologists (minimum 3-years’ experience, (blinded regarding physical features, clinical examinations, ultrasound examinations, and MRI examinations)) of the institute.

**Fig. 1:** Histopathology of the temporal artery (arrow shows giant cell arteritis). Magnification view*: 100; magnification bar: 25* μm

### Ultrasound examinations

Ultrasound examinations of longitudinal and transverse views of both (right and left) temporal arteries, both (right and left) axillary arteries including branches, both (right and left) parietal ramus, both (right and left) proximal frontal ramus, and both (right and left) distal frontal ramus had been taken by ultrasound equipment (Esaote SpA, Genoa, Italy) using an LA 424 linear probe at 13 MHz frequency (Esaote SpA, Genoa, Italy for B-Mode) and 10 MHz frequency (Esaote SpA, Genoa, Italy for color Doppler). The depth of ultrasound was 1.5 cm for temporal arteries, axillary arteries including branches, parietal ramus, and proximal frontal ramus. That for distal frontal ramus was 2.5 cm (Fig. 2) [15]. Ultrasound examinations had performed by ultra-sonographers (minimum 3-years’ experience, blinded regarding physical features, clinical examinations, temporal artery biopsy examinations, and MRI examinations) of the institute.

RETRACTED

**Fig. 2:** Detailed process flowchart of ultrasound examinations

### MRI examinations

MRI examinations of longitudinal and transverse views of both (right and left) temporal arteries, both (right and left) axillary arteries including branches, both (right and left) parietal ramus, both (right and left) proximal frontal ramus, and both (right and left) distal frontal ramus had been taken by 3 T Magnetom Skyra MRI equipment (Siemens, Erlangen, Berlin, Germany) with a 20-channel head coil (Siemens, Erlangen, Berlin, Germany). Diffusion-weighted images (a single-shot, spin-echo, and echo-planar), fast saturated T1 W1 (spin-echo sequence), and angiography were recorded before and after administration of 16 mL of gadolinium. Arterial segments were evaluated in cross-sectional views. Axillary arteries including branches and occipital artery were evaluated for 3 cm or more in length (Fig. 3) [12]. MR images had performed by radiologists (minimum 3-years’ experience, blinded regarding physical features, clinical examinations, temporal artery biopsy examinations, and ultrasound examinations) of the institute.

**Fig. 3:** Detailed process flowchart of magnetic resonance imaging examinations

### Image analysis

Images were uploaded in RadiAnt DICOM Viewer, version 4.9.15 Beta (Mediant, Maciej Frankiewicz, Poznan, Poland).

At least 1.5 mm swelling of the homogeneous wall was considered as vasculitis (Fig. 4). If artery lumen was 50% of the original in color Doppler for non-homogeneous walls, was considered as stenotic (Fig. 5) and if the ultrasound was unable to describe the color of non-homogeneous artery lumen then it was considered as occluded (Fig. 6). A halo (an eccentric or circumferential hypoechoic ring) around the vessel wall (Fig. 7), vasculitis, stenotic, or occluded either of temporal arteries, axillary arteries (including branches), parietal ramus, proximal frontal ramus, or distal frontal ramus was considered as giant cell arteritis [13]. Ultrasound images were analyzed by ultra-sonographers of the institute with a minimum of 3 years of experiences in ultrasound image analysis (blinded regarding physical features, clinical examinations, temporal artery biopsy examinations, and MRI examinations).

RETRACTED

**Fig. 4:** Ultrasound image of the temporal artery wall. **a**. Pictorial presentation of the temporal artery wall (normal and swelled). **b**. Color doppler longitudinal view of the swelled temporal artery wall (1.5 cm inflammation)

**Fig. 5:** Pictorial presentation of stenotic (artery lumen was 50% of the original)

**Fig. 6:** Pictorial presentation of the occluded artery (ultrasound was unable to describe the color of the artery lumen)

**Fig. 7:** Ultrasound image of an eccentric or circumferential hypoechoic ring around the temporal artery wall **a**. B-Mode longitudinal view of the temporal artery wall with a halo. **b**. Pictorial presentation of the temporal artery wall with a halo. The arrow shows halo

Mural enhancement and mural thickening were used as evaluation criteria for MR images analysis (Fig. 8). If at least one of ten different MR images either of temporal arteries, axillary arteries (including branches), parietal ramus, proximal frontal ramus, or distal frontal ramus had mural thickening of 0.6 mm or more and significant mural enhancement was considered as giant cell arteritis [16]. MRI was analyzed by radiologists of the institute with a minimum of 3 years of experiences in MR image analysis (blinded regarding physical features, clinical examinations, temporal artery biopsy examinations, and ultrasound examinations).

**Fig. 8:** Diagnosis of giant cell arteritis by magnetic resonance image **a**. Pictorial presentation of mural thickening. **b**. Magnetic resonance image of a longitudinal view of the temporal artery. The arrow shows mural thickening

### Beneficial score analysis

Decision curve analysis was applied to get a beneficial score for selected diagnostic modalities as per Eq. 1 and 2 [17]:

1 $$ \mathrm{Beneficialscore}=\frac{\mathrm{Truepositivegiantcellarteritisdetected}}{\mathrm{Numbersofpatientsenrolled}}-\left(\frac{\mathrm{Falsepositivegiantcellarteritisdetected}}{\mathrm{Numbersofpatientsenrolled}}\times \mathrm{Riskofoverdiagnosisandovertreatment}\right) $$

2 $$ \mathrm{Risk}\ \mathrm{of}\ \mathrm{overdiagnosis}\ \mathrm{and}\ \mathrm{overteratment}=\frac{\mathrm{Level}\ \mathrm{of}\ \mathrm{confidence}\ \mathrm{above}\ \mathrm{which}\ \mathrm{patients}\ \mathrm{were}\ \mathrm{put}\ \mathrm{on}\ \mathrm{glucocorticoid}\ \mathrm{a}\mathrm{s}\ \mathrm{a}\ \mathrm{precaution}\ }{1-\mathrm{Level}\ \mathrm{of}\ \mathrm{confidence}\ \mathrm{above}\ \mathrm{which}\ \mathrm{patients}\ \mathrm{were}\ \mathrm{put}\ \mathrm{on}\ \mathrm{glucocorticoid}\ \mathrm{a}\mathrm{s}\ \mathrm{a}\ \mathrm{precaution}\ } $$

RETRACTED

### Cost analysis

Physician charges for physical and clinical features examinations, to perform biopsies following histopathology, ultrasound findings, and MRI examinations [1] were collected from patients’ record of the institute(s) and pharmacy.

### Statistical analysis

InStat, version Window, GraphPad Software, San Diego, CA, USA was used for statistical analysis. The interobserver agreement was derived by Cohen k test (value of k ≥ 0.80 considered as outstanding agreement and a value of 0.8 > k ≥ 0.60 was considered as good agreement) according to Landis and Koch [16]. Constant data were analyzed by the Chi-square test of Independence [12]. Continuous variables were analyzed by one-way analysis of variance (ANOVA) or Wilcoxon’s signed rank test [11]. The results were considered significant at 99% of confidence level.

## Results

### Characteristics of study participants

During 15 March 2016 to 31 December 2018, a total of 1000 patients were referred to the First Hospital of Lanzhou University, China by rheumatologists, ophthalmologist, and neurologists as a suspected disease of giant cell arteritis. Among them, 5 patients had already diagnosed with giant cell arteritis and 15 patients had received glucocorticoid treatment. Therefore, they were excluded from the analysis (Fig. 9).

**Fig. 9:** Flow chart of the analysis

Data of 980 patients were included in the study. Mean age of enrolled patients were 61.12 ± 6.56 years. 48% of patients were females and 52% of patients were males. The other demographic and clinical characteristics of enrolled patients are reported in Table 1. Patients had one or more symptoms at the time of enrollment. Therefore, consultants had diagnosed as suspected giant cell arteritis.

**Table 1:** The demographic, social, and clinical characteristics of enrolled patients

Characters		Value
Patients enrolled in the cohort		980
Age (years)	Minimum	51
	Maximum	79
	Mean ± SD	61.12 ± 6.56
Gender	Male	474(48)
	Female	506(52)
Fever		102(10)
Asthenia		15(2)
Anorexia		19(2)
Recent visual impairment		211(22)
C-reactive protein level < 5 mg/dL		245(25)
Jaw or tongue claudication		311(32)
Shoulder girdles		345(35)
Pain in the hip		411(42)
Abnormal liver functions		245(25)
Temporal artery tenderness		311(32)
Weight loss, > 2 kg		189(19)
Erythrocyte sedimentation rate (mm/h)		56.47 ± 5.47
Ethnicity	Ha Chinese	978(99.8)
	Tibetan	01(0.1)
	Mongolian	01(0.1)
History of smoking	Non-smokers	325(33)
	Previous smokers	446(46)
	Current smokers	209(21)

Constant data are represented as a number (percentage) and continuous data are represented as mean ± SD

RETRACTED

### Interobserver agreement

A total of seven physicians, five ultra-sonographer, and six radiologists were involved in the interpretations of physical and clinical features, image analysis of ultrasound and MRI respectively. Interobserver agreement for the physical and clinical features interpretations was outstanding (k = 0.83), for image analysis of ultrasound examinations was good (k = 0.62), and for image analysis of MRI examinations was good (k = 0.67) respectively (Table 2).

**Table 2:** Interobserver agreement

Parameters	Diagnostic modalities			
	Physical and clinical features	Temporal artery biopsy	Ultrasound	Magnetic resonance imaging
Observers involved	7	4	5	6
Specialty	Neuro physicians, ophthalmologists, physician, pathologists	Pathologists	Ultra-sonographer	Radiologist
Tools	Questionaries’ and laboratory tests	4 cores	B-mode and color doppler	DWI and T1WI
Criteria for positive giant cell arteritis	The new type of localized head pain, and claudication of jaw or tongue	Visualization of giant cell in histopathology	Halo, vasculitis, stenotic, or occluded	Mural thickening ≥0.6 mm and significant mural enhancement
k-value	0.83	0.63	0.62	0.67

k ≥ 0.80: outstanding agreement, 0.8 > k ≥ 0.60: good agreement

All observers had minimum 3-years of experience

### Diagnostic parameters

More numbers of true positive giant cell arteritis cases (650 vs. 643) and true negative giant cell arteritis cases (100 vs. 50, *p* < 0.0001) were reported in case of physical and clinical features examinations following ultrasound detection than physical and clinical features examinations following temporal artery biopsy examinations. Also, less numbers of false positive giant cell arteritis cases (45 vs. 127, *p* < 0.0001) and false negative giant cell arteritis cases (15 vs. 35, *p* = 0.007) were reported in case of physical and clinical features examinations following ultrasound detection than physical and clinical features examinations following temporal artery biopsy examinations. Sensitivity was in the order of MRI examinations > physical and clinical features examinations following temporal artery biopsy examinations > physical and clinical features examinations following ultrasound detection but accuracy were in the order of MRI examinations > physical and clinical features examinations following ultrasound detection > physical and clinical features examinations following temporal artery biopsy examinations. There was no significant difference for true negative results between MRI and physical and clinical features examinations following ultrasound detection (140 vs. 100, *p* = 0.007, Table 3).

RETRACTED

**Table 3:** Diagnostic parameters of adopted modalities

Parameters of giant cell arteritis	Diagnostic modalities examinations										
	MRI	PC		TAB		PC + TAB		Us		PC + Us	
		Value	^*^ *p*	Value	^*^ *p*	Value	^*^ *p*	Value	^*^ *p*	Value	^*^ *p*
Patients enrolled	980	980		980		980		980		980	
True positive	840(86)	350(36)	< 0.0001	400(41)	< 0.0001	643(65)	< 0.0001	385(39)	< 0.0001	650(66)	< 0.0001
True negative	140(14)	40(4)	< 0.0001	50(5)	< 0.0001	50(5)	< 0.0001	45(5)	< 0.0001	100(10)	0.007
False positive	0(0)	290(30)	< 0.0001	270(28)	< 0.0001	127(13)	< 0.0001	46(5)	< 0.0001	45(5)	< 0.0001
False negative	0(0)	100(10)	< 0.0001	85(9)	< 0.0001	35(4)	< 0.0001	15(2)	0.0003	15(2)	< 0.0001
Inconclusive	0(0)	200(20)	< 0.0001	175(18)	< 0.0001	125(13)	< 0.0001	489(50)	< 0.0001	170(17)	< 0.0001
Sensitivity	1	0.8	< 0.0001	0.82	< 0.0001	0.87	< 0.0001	0.5	< 0.0001	0.83	< 0.0001
Accuracy	1	0.4	< 0.0001	0.46	< 0.0001	0.71	< 0.0001	0.44	< 0.0001	0.77	< 0.0001

*MRI* Magnetic resonance imaging

*PC* Physical and clinical features examinations

*TAB* Temporal artery biopsy examinations results

*Us* Ultrasound examinations results

Continuous variables are represented as mean and constant variables are represented as number (percentage)

Constant data were analyzed by the Chi-square test of Independence

The results were considered significant if *p* < 0.01

^*^p-value comparison with respect to MRI examinations

### The risk of overdiagnosis and overtreatment

The working area that detects giant cell arteritis at least one time for physical/ clinical features examinations following ultrasound detection and physical/ clinical features examinations following temporal artery biopsy examinations were 0–91% (high- and medium-risk giant cell arteritis patients) and 0–86% (high-risk giant cell arteritis patients) respectively. Above 91% (for low-risk giant cell arteritis patients) for ultrasound detection and above 86% (for low-and medium-risk giant cell arteritis patients) for temporal artery biopsy had the risk of overdiagnosis and overtreatment respectively (Fig. 10).

**Fig. 10:** Decision curve analysis. a: an area that detects high-risk giant cell arteritis at least one time, b: an area that detects medium-risk giant cell arteritis at least one time, c: an area that detects low-risk giant cell arteritis at least one time. Ultrasound images were analyzed by ultra-sonographers, magnetic resonance images were analyzed by radiologists, the physical and clinical features interpretations were performed by physicians, and the biopsies results were interpreted by pathologists (all evaluators had minimum 3 years of experiences)

RETRACTED

### Cost

Physical and clinical features examinations following ultrasound detection were less expensive method than physical and clinical features examinations following temporal artery biopsy examinations (14,023 ± 982 ¥/patient vs. 18,551 ± 1231 ¥/patient, *p* < 0.0001, Fig. 11).

**Fig. 11:** Cost Analysis of adopted diagnostic methods. Patients enrolled were 980 for all analyses. Data are presented as mean ± SD of all. Variables were analyzed by one-way ANOVA. The results were considered significant if *p* < 0.01.^*^less expensive method than physical and clinical features examinations following temporal artery biopsy examinations and also magnetic resonance imaging method

## Discussion

The prospective cohort study concluded that physical/ clinical features examinations following ultrasound detection had high accuracy (0.77 respect to MRI) and no risk of the overdiagnosis and overtreatment in the detection of high- and medium-risk giant cell arteritis in the enrolled patients. High accuracy is required in case of suspected giant cell arteritis [16] because corticosteroid treatment is the only effective treatment currently available for giant cell arteritis and corticosteroid therapy has bruising, cataracts and proximal weakness as treatment-emergent adverse effects [10]. The results of the study were in line with available studies [1, 11, 13, 15]. However, TABUL study enrolled only 381 patients and have used clinical features and physical examinations as ‘gold standard’ [1], case series study has enrolled only 46 patients and 6-month evaluation of the patients have used as ‘gold standard’ [11], and case-control study also enrolled only 176 patients but without ‘gold standard’ [13]. These available studies are full-filled the American College of Rheumatology (ACR) 1990 criteria for the diagnosis of giant cell arteritis [18] but do not highlight the overdiagnosis and overtreatment in giant cell arteritis. With respect to the results of the study, low-and medium-risk giant cell arteritis patients can have a risk of side effects due to systemic corticosteroid if they are diagnosed as giant cell arteritis by temporal artery biopsy examinations.

The study reported that ultrasound detection is non-invasive and cost-effective method than temporal artery biopsy examinations. The results of the study were parallel with those of TABUL study [1], a retrospective study [19], a consecutive case series [11], and a case report [15]. Giant cell arteritis has issues of personal, social care, and socioeconomic costs [20]. A biopsy would result in discomfort, bruising, bleeding, or infection at the site of the area [1]. To overcome the cost factor fast track pathway was introduced in 2012 [20, 21]. Factor fast track pathway reduce the risk of permanent visual impairment [7, 20] but fast track pathway requires high awareness of general practitioners [7], which is difficult to achieve in developing countries. Additionally, in China, the cost of fast track pathway is around 16,000 ¥ (greater than ultrasound examinations) to diagnose giant cell arteritis. Also, fast track pathway is also relaid on ultrasound detection [22] but in fast track pathway ultrasound examination is carried out by rheumatologist not by specialized ultra-sonographer(s) [23]. In respect to socioeconomic factors of suspected giant cell arteritis patients, conventional ultrasound detection is a suitable diagnostic modality for the detection of giant cell arteritis in Chinese patients.

RETRACTED

Large numbers of false negative giant cell arteritis patients were reported by temporal artery biopsy examinations than ultrasound examinations (85 vs. 15, *p* < 0.001). The results of the study were parallel with those of TABUL study [1] and prospective multicenter trial [16]. The possible justification for the same was that there would be a patchy inflammation in the artery wall, samples of biopsy were taken from the area where no inflammation [11], or incidence of the giant cell arteritis in the patients has seasonal variation (an environmental etiology) [10, 24, 25]. All in all, the diagnosis of giant cell arteritis is clinicians’ challenge.

The study reported that physical and clinical features examinations following ultrasound detection had minimal sensitivity. The results of the study were in line with TABUL study [1] but not in line with a consecutive case series [11]. The possible reason for that was ultra-sonographers had difficulties in capturing abnormalities in ultrasound images. Therefore, training is required for ultra-sonographers before scanning the patients. Also, technical standardization of ultrasound equipment, image acquisition, and probe settings are required. Additionally, MRI would be preferred diagnostic modality in patients, whose diagnosis remains disorganized even after ultrasound examination.

With reference to MRI, physical and clinical features examinations following ultrasound detection had fewer sensitivity and accuracy (*p* < 0.0001 for both) but no significant difference for true negative results (*p* = 0.007) and cost of diagnosis was also low (14,023 ± 982 ¥/per patient vs. 24,221 ± 1545 ¥/per patients, *p* < 0.0001). MRI has issues of availability [1]. Additionally, in physical and clinical features examinations following ultrasound do not involve ionizing radiation [13]. MRI has a low field of view and the contrast enhancement of walls of arteries would also be due to atherosclerotic plaques [12]. However, ultrasound can successful in discrimination of giant cell arteritis and atherosclerotic plaques [26]. Moreover, for the circle of Willis, the thin-walled intradural arteries do not show any mural enhancement and/or mural thickening under MRI [15, 27]. The MRI protocol is not specifically adjusted to depict mural inflammation of the superficial cranial arteries and to visualize the intradural arteries [12]. MRI has no ability to discriminate polyarteritis nodosa, systemic antineutrophilic cytoplasmatic antibody–positive vasculitis, and another inflammatory disease from giant cell arteritis [16]. However, Ultrasound has advantages of safety, availability, tolerability, and its high resolution of 0.1 mm [23]. Ultrasound of temporal and extracranial arteries also correlates well with MRI [13, 19]. Therefore, physical characters and clinical examinations following ultrasound finding is a suitable modality for the diagnosis of giant cell arteritis.

RETRACTED

Although the study was the large sample prospective study, there are several limitations of the study have reported, for examples, lack of follow-up data regarding treatment. More numbers of inconclusive results were reported for physical and clinical features examinations following ultrasound detection than physical and clinical features examinations following temporal artery biopsy examinations (170 vs. 125, *p* = 0.005). There are no predefined limits of ultrasound available for the diagnosis of giant cell arteritis in PR China by the ministry of the health department. Lower systemic inflammatory response [4], gender [3], age [10], and the history of smoking [4] have effects on prevalence of giant cell arteritis but the study did not evaluate such independent parameters in the analysis.

## Conclusion

Temporal artery biopsy is a useful technique for the detection of giant cell arteritis but it was a costly and expensive method. Also, it had the chances of overdiagnosis and overtreatment for low-and medium-risk giant cell arteritis. Physical and clinical features examinations following ultrasound detection are non-invasive, economical diagnostic modality, had high specificity, and no chances of overdiagnosis and overtreatment for high and medium-risk giant cell arteritis. The study recommended an ultrasound technique for diagnosis of patients with suspected giant cell arteritis.

## Data Availability

The datasets used and analyzed during the current study available from the corresponding author on reasonable request.

## Abbreviations

ANOVA: Analysis of variance
ESR: Erythrocyte sedimentation rate
MRI: Magnetic resonance imaging
STROBE: The strengthening the reporting of observational studies in epidemiology
